The article "Abdominal Aortic Aneurysm: An Overlooked Etiology of Low Back Pain" was retracted in 2024. Reasons: false authorship; unreliable results or conclusions; no approval from an author; concerns about the authorship.

# Abdominal Aortic Aneurysm: An Overlooked Etiology of Low Back Pain

**DOI:** 10.7759/cureus.18587

**Published:** 2021-10-07

**Authors:** Saad M Alabdullatif, Mohammed H Alajwad, Mishal F Kareemah, Israa A Almaghasilah, Abdullah M Alsaedan, Nawaf T Alenazi, Abdullah S Alshaibani, Mohammad K Abusaleh, Lojain M Maawadh, Ahmad A Alsolaiman, Malak Alshammari

**Affiliations:** 1 College of Medicine, Imam Abdulrahman Bin Faisal University, Dammam, SAU; 2 Pediatrics, Maternity and Children Hospital, Dammam, SAU; 3 College of Medicine, Umm Al Qura University, Mecca, SAU; 4 College of Medicine, Shaqra University, Shaqraa, SAU; 5 College of Medicine, Alfaisal University, Riyadh, SAU; 6 College of Medicine, Vision Colleges, Riyadh, SAU

**Keywords:** elderly patients, endovascular surgical repair, low back pain, abdominal aortic aneurysms, case report

## Abstract

Low back pain is very common and the vast majority of cases are related to non-specific etiologies. Low back pain due to serious pathologies is very rare. We present the case of a 66-year-old man with progressively worsening low back pain. His past medical history was remarkable for poorly controlled hypertension, diabetes mellitus, and dyslipidemia. He had several visits to the outpatient clinics and was diagnosed as having low back pain due to musculoskeletal etiology. He was prescribed multiple oral non-steroidal anti-inflammatory drugs and underwent multiple sessions of physiotherapy. However, his condition progressed, and did not show any clinical improvement. He underwent a plain radiograph of the lumbosacral spine which revealed decreased intervertebral disc spaces with multiple osteophytes. However, aneurysmal dilatation of the abdominal aorta was noted with atheromatous calcification. Computed tomography angiography confirmed the diagnosis of abdominal aortic aneurysm. The patient underwent endovascular repair of the aneurysm. The patient had complete resolution of his low back pain and remained symptom-free after six months of follow-up. The present case highlighted that those common presentations such as low back pain can be indicative of serious underlying pathology. Early diagnosis and management of abdominal aortic aneurysms can improve the prognosis and survival.

## Introduction

Low back pain is very common with a lifetime prevalence of approximately 85% [1]. Importantly, low back pain is considered the leading cause of years of life lost due to disability according to the Global Burden of Disease Study in 2016 [2]. The vast majority of low back pain is related to non-specific mechanical etiologies. In most cases, the episode of low back pain is self-limiting. Although rare, the patient should be comprehensively evaluated for possible serious etiologies. Low back pain due to serious pathologies accounts for less than 1% of all cases [3]. Such pathologies include cauda equina syndrome, metastatic cancer, spinal epidural abscess, vertebral osteomyelitis. We report the case of an elderly man presenting with low back pain. After thorough investigation, the etiology of low back pain was due to abdominal aortic aneurysm, which is an unusual etiology of back pain.

The article "Abdominal Aortic Aneurysm: An Overlooked Etiology of Low Back Pain" was retracted in 2024. Reasons: false authorship; unreliable results or conclusions; no approval from an author; concerns about the authorship.

## Case presentation

We present the case of a 66-year-old man who presented to the emergency department with worsening low back pain. He reported that he started to experience this pain in the last year, but it has been gradually increasing in severity. The pain was non-radiating, constant, and was noted related to posture or movement. The patient could not identify any exacerbating factors for his pain, but he stated that the standard analgesic medications become not fully effective for his pain. He rated the pain as 7 out of 10 in severity and this pain started to affect his quality of daily living. There was no history of preceding trauma. The pain was not associated with weakness or numbness in the lower extremities and there were no disturbances in the urinary or fecal continence. The patient did not experience weight loss, decreased appetite, or night sweats. He reported visiting several outpatient clinics for his pain, which was diagnosed as mechanical low back pain. He was prescribed several oral non-steroidal inflammatory drugs and underwent several sessions of physiotherapy.

The past medical history of the patient was remarkable for long-standing hypertension, diabetes mellitus, and dyslipidemia. He was receiving perindopril 10 mg once daily, atorvastatin 20 mg once daily, and metformin 800 mg twice daily. However, his conditions were not well-controlled due to non-adherence to lifestyle modification and pharmacologic treatments. He had a history of laparoscopic cholecystectomy performed after an attack of acute cholecystectomy. He was a smoker with a 30 pack-year history of smoking. He did not drink alcohol. He worked as a school teacher. His family history was non-contributory.

Upon examination, the patient was alert, conscious, and oriented. He looked in mild distress due to the pain. His vital signs were as follows: pulse rate of 90 bpm, blood pressure of 146/86 mmHg, respiratory rate of 13 bpm, and temperature of 37.1℃. Examination of the lumbar spine revealed tenderness along the vertebrae with mild restriction in the range of motion due to the pain. Neurological examination of the lower limbs showed normal tone and power bilaterally with normal reflexes. The cardiorespiratory examination was normal. Initial laboratory investigation revealed a hemoglobin level of 14.2 g/dL, a leukocyte count of 5600/µL, and a platelet count of 350,000/µL.

The article "Abdominal Aortic Aneurysm: An Overlooked Etiology of Low Back Pain" was retracted in 2024. Reasons: false authorship; unreliable results or conclusions; no approval from an author; concerns about the authorship.

In view of the aforementioned clinical information, the initial diagnosis was low back pain due to mechanical etiology. However, considering the longstanding history of the patient, a lumbosacral radiograph was performed. It revealed decreased intervertebral disc spaces with multiple osteophytes. Importantly, there was evidence of aneurysmal dilatation of the lower abdominal aorta with atheromatous calcification (Figure 1). Subsequently, the patient underwent computed tomography angiography which confirmed the diagnosis of abdominal aorta aneurysm, measuring 8.2 in the maximum diameter (Figure 2).

**Figure 1:** Plain Radiograph Frontal (A) and lateral (B) plain radiograph images of the lumbosacral spine demonstrating aneurysmal dilatation of the lower abdominal aorta with atheromatous calcification (arrows).

**Figure 2:** Computed Tomography Axial computed tomography angiography demonstrating aortic aneurysm (arrow) with circumferential thrombus.

The patient was referred to the vascular surgery team due to the risk of rupture. The patient underwent endovascular treatment of the aneurysm. The procedure was performed successfully with no post-operative complications. The patient had complete resolution of his pain. After six months of follow-up, the patient had major satisfaction as he remained symptom-free since the procedure.

## Discussion

We presented the case of an elderly man with an abdominal aortic aneurysm presenting with a one-year history of low back pain that was managed conservatively with oral analgesics and physiotherapy. An abdominal aortic aneurysm is defined as an abnormal focal dilatation of the abdominal aorta, which is a common and potentially life-threatening condition.

It is crucial to recognize the clinical manifestations of low back pain that may suggest a non-mechanical etiology of the low back pain that warrants further investigation and evaluation. For example, in the present case, the patient could not identify any aggravating or relieving factors for the pain and it was not related to posture. Comprehensive history taking is crucial to rule out the serious pathologies of low back pain with a greater emphasis on the constitutional symptoms. A plain lumbosacral radiograph is a relatively cheap and widely available investigation that could provide help in ruling out serious pathologies. The current case suggests that physicians should have a low threshold in requesting a plain radiograph for evaluating back pain of unknown etiology.

The majority of patients with an abdominal aortic aneurysm are asymptomatic and are diagnosed incidentally on imaging. When symptomatic, an abdominal aortic aneurysm usually presents with abdominal pain, flank pain, and thromboembolic events leading to limb ischemia. An untreated ruptured abdominal aortic aneurysm is fatal. The mortality rate of ruptured abdominal aortic aneurysms for patients reaching the hospital exceeds 50% [4]. Hence, the identification of patients with an unruptured abdominal aortic aneurysm can be life-saving.

The article "Abdominal Aortic Aneurysm: An Overlooked Etiology of Low Back Pain" was retracted in 2024. Reasons: false authorship; unreliable results or conclusions; no approval from an author; concerns about the authorship.

Several factors have been identified as risk factors for the development of abdominal aortic aneurysm and its rupture. Male patients and advanced age are the most significant factors. The abdominal aortic aneurysm is more prevalent among the white population and those having a family history. Having other large vessel aneurysms is also a risk factor for abdominal aortic aneurysms [5].

Aneurysm repair is indicated in all symptomatic patients and those who have aneurysmal dilatation larger than 5.5 cm. The repair can be accomplished using an open or endovascular technique. In the present case, the endovascular approach was used as the patient could be at higher operative risk. Close observation is recommended for patients with abdominal aortic aneurysms below the size criteria for intervention. Smoking cessation should be strongly advised as it is the only factor that was found to slow the progression of the aneurysm [5].

## Conclusions

The present case highlighted those common presentations such as low back pain can be indicative of serious underlying pathology. Clinicians should remain alert and maintain a high index of suspicion for abdominal aortic aneurysms in the population at risk. Early diagnosis and management of abdominal aortic aneurysms can improve the prognosis and survival.
